# The novel long non-coding RNA LATS2-AS1-001 inhibits gastric cancer progression by regulating the LATS2/YAP1 signaling pathway via binding to EZH2

**DOI:** 10.1186/s12935-020-01285-w

**Published:** 2020-05-29

**Authors:** Dan Sun, Ying Wang, Huan Wang, Yan Xin

**Affiliations:** 1 Laboratory of Gastrointestinal Onco-Pathology, Cancer Institute & General Surgery Institute, The First Affiliated Hospital of China Medical University, No. 155 Nanjing North Street, Heping District, Shenyang, 110001 China; 2 Department of Oncology, Hanzhong Central Hospital, Hanzhong, 723000 China

**Keywords:** Long non-coding RNA, Large tumor suppressor 2/LATS2, Yes-associated protein 1/YAP1, Enhancer of zeste homolog 2/EZH2, Gastric cancer

## Abstract

**Background:**

To explore the expression pattern and role of the novel long non-coding RNA LATS2 antisense transcript 1 (LATS2-AS1-001) in gastric cancer (GC).

**Methods:**

qRT-PCR was applied to evaluate LATS2-AS1-001 expression and correlation with LATS2 in GC. In vitro experiments were performed to investigate the role of LATS2-AS1-001 in GC cells. RNA immunoprecipitation (RIP) was performed to assess the interaction between EZH2 and LATS2-AS1-001. LATS2/YAP1 signaling pathway proteins were detected by immunoblot. Oncomine and KMPLOT data analysis was conducted to assess the prognostic value of YAP1 in GC.

**Results:**

Decreased expression levels of LATS2-AS1-001 and LATS2 were confirmed in 357 GC tissues compared with the normal mucosa. A strong positive correlation between LATS2-AS1-001 and LATS mRNA expression was found in Pearson Correlation analysis (r = 0.719, P < 0.001). Furthermore, ROC curve analysis revealed areas under the curves for LATS2-AS1-001 and LATS2 of 0.7274 and 0.6865, respectively (P < 0.001), which indicated that LATS2-AS1-001 and LATS could be used as diagnostic indicators in GC. Moreover, ectopic expression of LATS2-AS1-001 decreased cell viability, induced G0/G1 phase arrest, and inhibited cell migration and invasion in GC cells. Mechanistically, overexpressing LATS2-AS1-001 upregulated LATS2 and induced YAP1 phosphorylation via binding to EZH2. Oncomine and KMPLOT database analysis demonstrated YAP1 was highly expressed in human GC samples, and high YAP1 expression predicted poor patient prognosis in GC.

**Conclusion:**

This study revealed that lncRNA LATS2-AS1-001 might serve as a potential diagnostic index in GC and act as a suppressor of GC progression.

## Background

Despite its recent decline, gastric cancer (GC) is considered the third leading cause of cancer-related death around the world, following lung and liver cancers [1]. Its incidence vary geographically, with the highest rates recorded in Eastern Asian countries, including Korea, Mongolia, Japan and China; in these nations GC patients usually have poor prognosis due to unapparent early symptoms and imperceptible invasion and metastasis [2, 3]. Therefore, there is an urgent need for identifying early biomarkers of GC and exploring their potential molecular mechanisms.

Long non-coding RNAs (lncRNAs) are RNA molecules longer than 200 nucleotides, which do not have the ability to produce proteins due to loss of open reading frames. Most lncRNAs result from transcription by RNA polymerase II and polyadenosinic acid [4, 5]. According to genomic location and context, lncRNAs are classified into four groups, including intergenic, intronic, sense and antisense lncRNAs [6]. LncRNAs, which were previously considered “noise” due to lack of protein-encoding capability, have been shown to participate in multiple biological processes, including transcription regulation, post-transcription regulation, cell cycle and apoptosis, cancer invasion and metastasis, and stem cell pluripotency [6–8]. Moreover, lncRNAs have been shown to be differently expressed in malignant cells and matched normal tissues, e.g., in breast cancer [9], non-small lung cancer [10], colorectal cancer [11] and liver cancer [12]. Furthermore, recent studies have suggested that various lncRNAs may function as an oncogene or a tumor suppressor possibly by regulating cell proliferation, cell cycle, apoptosis, migration and invasion through interaction with Notch, mTOR, NF-κB and Wnt signaling pathways in GC [13–15].

Large tumor suppressor 2 (LATS2), located on chromosome 13q12.11, is the core serine/threonine kinase of the Hippo tumor-suppressive signaling pathway. LATS2 regulates the cell fate by modulating the functions of the downstream Hippo effectors YAP/TAZ [16]. Studies have suggested that the LATS2 signaling pathway interacts with P53, estrogen signaling, and the Ras and Akt network, thus playing important roles in regulating cell proliferation, cell cycle and apoptosis, and cell invasion and migration in various carcinomas [17, 18]. LncRNA LATS2 antisense 1 (LATS2-AS1-001) is a 632 bp-long lncRNA located in the 21005157–21018122 region of chromosome 13. Accumulating evidence indicates that antisense transcripts, especially non-coding RNAs, might regulate sense genes [19]. LATS2 expression is considered a good prognostic factor in GC [20]. Nevertheless, to the best of our knowledge, the expression and effects of LATS2-AS1-001 in human tumors have not been investigated to date.

Enhancer of zeste homolog 2 (EZH2) has been reported in various carcinomas [21, 22]. EZH2 participates in tumor proliferation, migration and metastasis. Previous studies have demonstrated that long non-coding RNAs play vital roles in various tumors via EZH2 [23, 24]. However, the interaction between LATS2-AS1-001 and EZH2 has not been explored.

In present study, we examined the expression of LATS2-AS1-001 and its neighboring gene LATS2 in GC specimens, and analyzed the associations of their expression levels with clinicopathological features. Subsequent functional experiments were conducted by overexpressing LATS2-AS1-001. RNA immunoprecipitation (RIP) was performed to assess the interaction between LATS2-AS1-001 and EZH2. We hypothesized that LATS2-AS1-001 might play a suppressor role in GC progression by regulating the LATS2/YAP1 signaling pathway via binding to EZH2.

## Materials and methods

### Patient sample collection

A total of 357 fresh human GC tissue samples and matched normal adjacent tissue (distance from gastric cancer ≥ 5 cm) specimens were collected from patients who underwent cancer resection in The First Hospital of China Medical University between 2007 and 2016. These fresh samples were immediately snap frozen in liquid nitrogen after operation. The clinicopathological data recorded included age, gender, tumor size, Lauren’s type and WHO type (Table 1). TNM stages were evaluated based on the UICC (Union for International Cancer Control)/AJCC (American Joint Committee on Cancer) Clinical Practice Guidelines for Gastric Cancer (7th Edition).

**Table 1:** Correlation between LATS2-AS1-001 expression and clinicopathological features of gastric cancer

Groups	n	LATS2-AS1-001 expression		P
		High	Low	
Gender				0.646
Male	267	81	186	
Female	90	25	65	
Age (year)				0.220
≥60	202	59	143	
< 60	155	47	108	
Tumor size				0.167
≥ 5	252	70	182	
< 5	105	36	69	
Borrmann’s types				0.394
Bor.I + II	30	11	19	
Bor.III + IV	327	95	230	
WHO’s histological types				0.448
Papillary adenocarcinoma	6	3	3	
Tubular adenocarcinoma				
Well differentiated	10	2	8	
Moderately differentiated	80	25	55	
Poorly differentiated	219	67	152	
Signet ring cell adenocarcinoma	27	6	21	
Mucinous adenocarcinoma	15	3	12	
Lauren’s types				0.905
Intestinal	96	30	66	
Diffuse	180	55	125	
Mixed	81	21	60	
Depth of invasion				0.568
T1 + 2	26	9	17	
T3 + 4	331	97	234	
Lymph node metastasis				0.282
N0	78	27	51	
N1–3	279	79	200	
Distant metastasis				0.968
M0	345	103	242	
M1	12	3	9	
TNM staging				*0.032*
I + II	100	38	62	
III + IV	257	68	189	

Significance of P < 0.05 is indicated in italic

The Clinical Research Ethics Committee of the First Affiliated Hospital of China Medical University approved this study. In addition, all participants provided written informed consent.

### Cell culture

The human immortalized normal gastric mucosa GES-1 and gastric carcinoma MGC803, BGC823, SGC-7901, MKN-45 and HGC27 cell lines were purchased from Shanghai GeneChem Co., Ltd and conserved in the Laboratory of China Medical University Gastrointestinal Oncopathology. The cell lines were cultured in RPMI 1640 (Hyclone, Thermo scientific, USA) supplemented with 10% fetal bovine serum (Hyclone, USA) in a humidified atmosphere containing 5% CO_2_ at 37 °C.

### RNA extraction and real-time PCR

EASYspin Plus kits purchased from Beijing Aidlab Biotechnologies (China) were used to isolate total RNA from the collected GC and matched normal adjacent tissue samples, as well as from cultured GES-1 and MGC803, BGC823, SGC-7901, MKN-45 and HGC27 cells, according to the manufacturer’s instructions. The obtained total RNA was reverse transcribed with the PrimeScript^®^ RT Master Mix (Takara). Forward and reverse primers were, respectively: LATS2-AS1-001, 5′-CTCTGGCACTCCTACT-3′ and 5′-CTGGACCTGAACCTAC-3′; LATS2, 5′-CTCTGGCACTCCTACT-3′ and 5′-CTGGACCTGAACCTAC-3′; YAP1, 5′-TACGATACAAGGCTGTTAGAGAG-3′ and 5′-TTGAGATGCATGCTTTGCATA C-3′; EZH2, 5′-GTGGAGAGATTA TTTCTCAAGATG-3′ and 5′-CCGACATA CTTCAGGGCATCAGCC-3′; GAPDH, 5′-GAAGGTGAAGGTCGGAGTC-3′ and 5′-GAAGATGG TGATGGGATTTC-3′. The data were analyzed by the 2^−∆∆Ct^ method, using GAPDH for normalization.

### Western blot

Harvested cells and GC tissue samples were lysed in lysis buffer. BCA assay Kit (Beyotime, China) was used to quantify total protein concentration. Equal amounts of Total protein were separated by 10% SDS-PAGE and transferred onto polyvinylidene fluoride (PVDF) membranes. The membranes were blocked and incubated overnight at 4 °C with the following specific primary antibodies: rabbit polyclonal anti-LATS2 antibody (1:200; Abcam, Cambridge, UK); rabbit monoclonal anti-YAP1 antibody (1:1000, Abcam); rabbit monoclonal anti-EZH2 antibody (1:1000, Abcam); rabbit monoclonal anti-phosphoS127-YAP1 antibody (1:1000, Abcam); rabbit monoclonal anti-Cyclin D1 antibody (1:1000; Cell signaling technology, USA); mouse monoclonal anti-GAPDH antibody (1:1000; Origene Co., Ltd., China). This was followed by incubation with goat anti-rabbit/mouse secondary antibodies (1:1000; Origene Co.). Finally, blots were detected by enhanced chemiluminescence and analyzed with the Quantity One software.

### Plasmids and transfection constructs

BGC823 and SGC7901 cell lines with low LATS2-AS1-001 expression were selected for transfection. Cells were transfected with the empty vector (control plasmid) and LATS2-AS1-001 plasmid (GeneChem Co.), respectively, with Lipofectamine™ 2000 (Invitrogen, USA), according to the manufacturer’s instructions. Stable cell lines were selected using G418. Untreated parental BGC823 and SGC7901 cells were assessed as baseline controls. LATS2-AS1-001 overexpression was evaluated by qRT-PCR. Cells transfected with the control plasmid were termed NC/BGC823 and NC/SGC7901 cells, respectively, while those transfected with the LATS2-AS1-001 plasmid were named AS1/BGC823 and AS1/SGC7901 cells, respectively.

### EZH2 silencing

The negative control (5′-UUCUCCGAACGUGUCACGUTT-3′) and a siRNA targeting EZH2 (5′-AAGACUCUGAAUGCAGUUGCU-3′) were synthesized by GenePharma Co., Ltd. (Shanghai, China). BGC823 cells were transfected with scramble and EZH2 siRNAs, respectively, using Lipofectamine 2000 (Invitrogen) according to the manufacturer’s instructions. After 48 h of transfection, the cells were collected for detecting the silencing efficiency by qRT-PCR.

### Cell counting kit (CCK-8)

CCK-8 was performed to assess cell viability. Briefly, 2 × 10^3^ cells were seeded in 96-well plates and incubated for 5 days. At each time point (every 24 h), 10 μl of sterile CCK-8 reagent (Solarbio, Beijing, China) was added to each well and incubated for another 3 h at 37 °C. Absorbance at 450 nm was determined on a microplate reader.

### Colony formation assay

A total of 2 × 10^2^ cells were seeded in 6-well plates and incubated for 12 days. The colonies were stained with 0.01% crystal violet, and the stained cells were counted. All experiments were performed in triplicate.

### Flow cytometry (FCM) for cell cycle and apoptosis analyses

The harvested cells were fixed with 70% ethanol overnight. They were then labeled with propidium iodide (PI) containing RNase, and incubated in the dark at 37 °C for 30 min. Cell cycle distribution after PI staining was analyzed by FCM. All experiments were run in triplicate.

### Wound healing assay

Cells in the exponential growth phase were harvested and seeded in a 60 mm dish. At 90% confluence, a line was drawn using a marker at the bottom of the dish, and a sterile 10 µl pipet tip was used to generate three separate wounds through the cells, perpendicular to the line. The cells were then gently rinsed in PBS and incubated in 5 ml of RPMI 1640 containing 2% FBS at 37 °C, in a humid environment with 5% CO2. Images of the scratches were taken under an inverted microscope at 10× magnification after 0, 24 and 48 h of incubation, respectively. The rate of wound healing was calculated to evaluate the cell migration ability.

### Transwell migration and invasion assays

24-well Transwell inserts (8.0 μm pore size, Corning, USA) were utilized to determine the migratory and invasive abilities of cells. In the cell migration assay, 2 × 10^4^ cells in serum free medium were placed in the upper chamber of a non-coated Transwell insert. Then, 500 µl complete culture medium containing 20% FBS was added to the lower chamber. The chambers were incubated for 24 h, and cells were fixed with 4% paraformaldehyde, stained with 1% crystal violet and analyzed under an inverted microscope. In the cell invasion assay, the transwell inserts were coated with Matrigel Basement membrane matrix (BD, USA) diluted with serum free medium before adding cells, and the plates were incubated for 48 h in a humid environment with 5% CO_2_ at 37 °C. The remaining steps were as described for the cell migration assay.

### Oncomine and KMPLOT database analysis

The available cancer microarray database Oncomine (http://www.oncomine.org) and Kaplan–Meier plotter (http://kmplot.com/analysis) were utilized to assess YAP1 expression and GC patient survival. The statistical analysis of YAP1 expression in DErrico Gastric Statistics was performed by the Student’s t-test. The entire analysis used 224894_at Reporter.

### RNA immunoprecipitation (RIP)

According to the instructions of the Magna RIP RNA-binding protein immunoprecipitation kit purchased from Millipore, the RIP assay was conducted to assess the interaction between EZH2 and LATS2-AS1-001. Total RNA was precipitated with anti-EZH2 antibody (Abcam, USA). Then, qRT-PCR was performed to measure the enrichment of immunoprecipitated RNAs.

### Statistical analysis

All quantitative data are mean ± SD. Comparisons between two groups were performed by the Student’s t-test. Multiple group comparisons were carried out by one-way ANOVA. All statistical analyses were performed with SPSS22.0 (IBM, New York, USA). Two-sided *P *< 0.05 was considered statistically significant.

## Results

### LATS2-AS1-001 and LATS2 are downregulated in gastric cancer

A total of three hundred and fifty-seven paired human GC and matched adjacent normal tissue samples were collected for LATS2-AS1-001 and LATS2 mRNA level detection. LATS2-AS1-001 mRNA levels were significantly decreased in GC (mean value = 0.04) compared with adjacent normal tissues (mean value = 0.07, Fig. 1a). Similarly, LATS2 mRNA amounts were significantly reduced in GC (mean value = 0.07) samples compared with paired normal tissues (mean value = 0.12, Fig. 1b).

**Fig. 1:** LATS2-AS1-001 and LATS2 expression levels are lower in GC compared with matched normal gastric mucosa. LATS2-AS1-001 and LATS2 expression levels were detected by qRT-PCR. Both LATS2-AS1-001 (**a**) and LATS2 (**b**) were downregulated in GC tissues compared with the normal gastric mucosa. The receiver operating characteristic (ROC) curves of LATS2-AS1-001 and LATS2 were constructed to assess the respective diagnostic values. Areas under curves for LATS2-AS1-001 (**c**) and LATS2 (**d**) were 0.7274 and 0.6865, respectively (P < 0.001). Correlation analysis was carried out to confirm a strong positive correlation between LATS2-AS1-001 and LATS2 mRNA expression levels (**e**, r = 0.719, P < 0.001). Western blot was performed to evaluate LATS2 protein expression in GC tissues. Consistent with mRNA expression, LATS2 protein levels were decreased in GC tissues compared with the normal gastric mucosa (**f**, **g**)

Furthermore, we determined whether LATS2-AS1-001 or LATS2 amounts were associated with clinicopathological factors. Both LATS2-AS1-001 and LATS mRNA levels in GC were only correlated with TNM stage (P < 0.05). There were no significant differences in LATS2-AS1-001 or LATS2 based on age, gender, tumor size, Borrmann’s type, WHO’s histological type and Lauren’s type (*P *> 0.05, Table 1 and Table 2).

**Table 2:** Correlation between LATS2 expression and clinicopathological features of gastric cancer

Groups	n	LATS2 expression		P
		High	Low	
Gender				0.165
Male	267	86	181	
Female	90	22	68	
Age (year)				0.797
≥ 60	202	60	142	
**< **60	155	48	107	
Tumor size				0.572
≥ 5	252	74	178	
**< **5	105	34	71	
Borrmann’s types				0.975
Bor.I + II	30	9	21	
Bor.III + IV	327	99	228	
WHO’s histological types				0.424
Papillary adenocarcinoma	6	3	3	
Tubular adenocarcinoma				
Well differentiated	10	5	5	
Moderately differentiated	80	23	57	
Poorly differentiated	219	68	151	
Signet ring cell adenocarcinoma	27	6	21	
Mucinous adenocarcinoma	15	3	12	
Lauren’s types				0.211
Intestinal	96	25	71	
Diffuse	180	60	120	
Mixed	81	23	58	
Depth of invasion				0.615
T1 + 2	26	9	17	
T3 + 4	331	99	232	
Lymph node metastasis				0.503
N0	78	26	52	
N1–3	279	82	197	
Distant metastasis				0.130
M0	345	102	243	
M1	12	6	6	
TNM staging				*0.047*
I + II	100	38	62	
III + IV	257	70	187	

Significance of P < 0.05 is indicated in italic

To further assess LATS2 protein expression, Western blot was performed. Consistent with the above mRNA results, the protein expression of LATS2 in GC was significantly decreased compared with normal mucosa tissues (Fig. 1f, g).

### LATS2-AS1-001 and LATS are potential diagnostic indicators in GC

ROC curve analysis showed areas under the curves for LATS2-AS1-001 and LATS2 of 0.7274 (P < 0.001) (Fig. 1c) and 0.6865 (P < 0.001) (Fig. 1d), respectively. These results indicated that LATS2-AS1-001 and LATS2 could be used as diagnostic indicators in GC. Additionally, a strong positive correlation between LATS2-AS1-001 and LATS mRNA levels was found in Pearson Correlation analysis (r = 0.719, P < 0.001, Fig. 1e). To sum up, these results suggested a potential positive correlation between LATS2-AS1-001 and LATS in GC.

### LATS2-AS1-001 is downregulated in BGC823 and SGC-7901 cells

The mRNA expression levels of LATS2-AS1-001 were detected in human gastric carcinoma (MGC803, BGC823, SGC-7901, MKN-45 and HGC27) and human immortalized normal gastric mucosa (GES-1) cells by qRT-PCR. The results showed that LATS2-AS1-001 mRNA levels were decreased in SGC7901 and BGC823 cells compared with GES-1 cells (Fig. 2a). To further examine its biological function in malignant cells, BGC823 and SGC7901 cells were transfected with a plasmid overexpressing LATS2-AS1-001. Efficient transfection and stable overexpression of LATS2-AS1-001 in BGC823 and SGC7901 cells were confirmed by qRT-PCR (Fig. 2b, c).

**Fig. 2:** Overexpression of LATS2-AS1-001 inhibits GC cell proliferation and colony formation. The expression pattern of LATS2-AS1-001 in GC cell lines is shown in **a**. Low expression of LATS2-AS1-001 was detected in BGC823 and SGC7901 cells compared with GES-1 cells. Ectopic expression of LATS2-AS1-001 in BGC823 and SGC7901 cell lines was analyzed by qRT-PCR (**b**, **c)**. The viability of BGC823 (**d**) and SGC7901 (**e**) cells after stable transfection was detected by CCK-8. Ectopic LATS2-AS-001 expression decreased GC cell proliferation after 5 days (*P < 0.05). The colony-formation assay demonstrated that LATS2-AS1-001 overexpression significantly suppressed proliferation in BGC823 (**f**) and SGC7901 (**g**) cells. Histograms of average clone numbers are shown in **h**, **i**, *P < 0.05

### Overexpression of LATS2-AS1-001 inhibits BGC823 and SGC7901 cell proliferation

CCK-8 and colony formation assay were performed to assess the effects of LATS2-AS1-001 overexpression on GC cell growth. Briefly, overexpression of LATS2-AS1-001 in AS1/BGC823 and AS1/SGC7901 cells obviously inhibited cell viability compared with the BGC823 (wild type), NC/BGC823, SGC7901 (wild type) and NC/SGC7901 groups after 5 days of incubation (*p *< 0.05) (Fig. 2d, e), while no significance was observed at 1 to 4 days.

Consistently, LATS2-AS1-001 overexpression impaired the colony formation abilities of AS1/BGC823 and AS1/SGC27 cells compared with the control groups after 12 days of continuous culture (P < 0.05, Fig. 2f, g). Specifically, 70 ± 4.58 and 81.33 ± 4.97 colonies, respectively, were formed in AS1/BGC823 and AS1/SGC27 groups, which showed reduced amounts compared with BGC823 (126 ± 8.89) and NC/BGC823 (123.66 ± 5.03), and SGC7901 (128.67 ± 19.00) and NC/SGC7901 (138.67 ± 5.13) (P < 0.05), respectively. These data revealed that LATS2-AS1-001 overexpression in AS1/BGC823 and AS1/SGC27 cells impaired their colony formation abilities (Fig. 2h, i).

### Overexpression of LATS2-AS1-001 induces cell cycle arrest in BGC823 and SGC7901 cells

To further investigate the effects of LATS2-AS1-001 on cell cycle distribution and apoptosis, GC cells were analyzed by flow cytometry. As shown in Fig. 3a, b, LATS2-AS1-001 overexpression significantly increased the percentage of G_0_/G_1_ phase cells, while decreasing those of S and G2/M phase cells in AS1/BGC823 and AS1/SGC27 cells (Fig. 3c, d). These results demonstrated that LATS2-AS1-001 overexpression induced G0/G1 cell cycle arrest and impeded GC cell proliferation.

**Fig. 3:** Overexpression of LATS2-AS1-001 induces G0/G1 cell cycle arrest. LATS2-AS1-001 overexpression in BGC823 (**a**) and SGC7901 (**b**) gastric cancer cells resulted in increased cell percentages in the G0/G1 phase. Accordingly, the percentages of S and G2/M phase cells were decreased. Data from three separate experiments are shown in **c**, **d**, *P < 0.05

## Overexpression of LATS2-AS1-001 suppresses migration and invasion in BGC823 and SGC7901 cells

Because LATS2-AS1-001 overexpression could inhibit GC cell proliferation, we further assessed the effect of LATS2-AS1-001 on cell invasion and migration. As shown in Fig. 4a–d, the scratch assay demonstrated that wound-healing rates were significantly decreased in AS1/BGC823 and AS1/SGC27 cells compared with the control groups from 24 to 48 h (P < 0.05). Additionally, migration in AS1/BGC823 and AS1/SGC27 cells after LATS2-AS1-001 overexpression was inhibited in a time-dependent manner. Transwell migration and invasion assays showed that obviously less AS1/BGC823 and AS1/SGC7901 cells migrated into and invaded the lower chamber of the Transwell system compared with the corresponding control groups (P < 0.05, Fig. 4e–h). These results indicated that overexpressing LATS2-AS1-001 might suppress the migratory and invasive abilities of gastric cancer cells.

**Fig. 4:** LATS2-AS1-001 overexpression inhibits GC cell migration and invasion in vitro. The scratch test revealed that BGC823 (**a**) and SGC7901 (**b**) cells overexpressing LATS2-AS1-001 had suppressed migration at 24 h and 48 h. The ratios of GC cells in the scratched area are shown in **c**, **d**, *P < 0.05. The numbers of BGC823 and SGC7901 cells overexpressing LATS2-AS1-001 were decreased compared with control values (original magnification, ×200, **e**, **f**). *P < 0.05. The numbers of invading cells in the AS1/BGC823 and AS1/SGC7901 groups were reduced compared with control values (original magnification, ×200, **g**, **h**), *P < 0.05

### LATS2-AS1-001 interacts with EZH2 and regulates LATS2 in GC

RIP was applied to assess whether LATS2-AS1-001 could bind to EZH2 using anti-EZH2 antibodies. The enrichment of LATS2-AS1-001 and EZH2 is shown in Fig. 5a, which demonstrated an interaction between LATS2-AS1-001 and EZH2. To evaluate the regulatory effect of EZH2 on LATS2, LATS2 mRNA was detected by qRT-PCR after EZH2 silencing in BGC823 cells. We found that LATS2 mRNA expression was significantly elevated after EZH2 knockdown (Fig. 5b, c). In addition, qRT-PCR demonstrated that LATS2 was upregulated following LATS2-AS1-001 overexpression in BGC823 and SGC7901 cells (Fig. 5d, e). These results suggested that LATS2-AS1-001 might interact with EZH2 and regulate the transcriptional expression of LATS2.

**Fig. 5:** LAST2-AS1-001 recruits EZH2 to upregulate LATS2, and promotes YAP1 phosphorylation. **a** RIP was performed to assess the interaction of LATS2-AS1-001 with EZH2. The enrichment of LATS2-AS1-001 with EZH2 was normalized to IgG. *P < 0.05. **b** The efficiency of EZH2 knockdown in BGC823 cells was assessed by qRT-PCR. **c** LATS2 mRNA levels were detected by qRT-PCR after EZH2 knockdown. LATS2 and YAP1 expression levels were measured by qRT-PCR and Western blot in BGC823 and SGC7901 cells overexpressing LAST2-AS1-001. The results showed that LATS-AS1-001 overexpression upregulated LATS2 (**d**, **e**, **h**), downregulated YAP1 (**f–h**) both at the mRNA and protein levels, and promoted YAP1 phosphorylation. In addition, the cell cycle related protein cyclin D1 was also downregulated after LATS-AS1-001 overexpression in GC cells (**h**)

### LATS2-AS1-001 overexpression promotes YAP1 phosphorylation and downregulates Cyclin D1 in GC cells

Notably, LATS2 serves as an important kinase protein in the Hippo/YAP signaling pathway and participates in the phosphorylation of the downstream effectors YAP and TAZ. To assess a potential interaction between LATS2 and YAP, Western blot was performed to assess phosphorylated and total YAP1 protein amounts, respectively, in BGC823 and SGC7901 cells transfected with vector and overexpressing LATS2-AS1-001 plasmids, respectively. As shown above, LATS2 mRNA and protein levels were significantly increased after LATS2-AS1-001 overexpression, while total YAP1 amounts were decreased both at the mRNA and protein levels (Fig. 5f–h). Meanwhile, phosphorylated YAP1 protein levels were elevated in BGC823 and SGC7901 cells transfected with the LATS2-AS1-001 plasmid (Fig. 5h). These results suggested that LATS2-AS1-001 could promote YAP1 phosphorylation by activating LAST2.

In addition, considering that LATS2-AS1-001 overexpression inhibited GC cell proliferation and induced G0/G1 phase arrest, the cell cycle protein Cyclin D1 was detected by Western blot. As shown in Fig. 5h, cyclin D1 expression was obviously decreased after LATS2 overexpression.

### YAP1 mRNA expression is significantly increased in GC tissues, and high YAP1 amounts predict poor patient prognosis in GC

Based on an Oncomine database analysis, YAP1 transcription levels were significantly elevated in GC tissues compared with the normal mucosa in DErrico Gastric datasets. Specifically, YAP1 was upregulated in GC types, including gastric intestinal adenocarcinoma, diffuse gastric adenocarcinoma and gastric mixed adenocarcinoma compared with the gastric mucosa (fold changes of 1.979 [P < 0.001], 1.650 [P < 0.001] and 2.089 [P < 0.01], respectively, Fig. 6a–d). To further investigate the relationship between YAP1 expression and prognosis, KMPLOT analysis was conducted in 876 GC patients. The results showed that YAP1 overexpression was closely related to poor overall survival (OS) and reduced first progression (FP) time in GC patients. Median OS in the high YAP1 expression group (35.9 months) was shorter than that of the low YAP1 expression cohort (63.7 months). Median FP time in the high YAP1 expression group was 25.3 months, which was also shorter than that of patients lowly expressing YAP1 (80.1 months). In agreement, high expression of YAP1 was an independent predictor of poor prognosis in terms of OS (HR = 1.31, P = 0.015) and FP (HR = 1.53, P = 0.003) in GC (Fig. 6e–f). These findings were consistent with our previous studies [25–27], which revealed that YAP1 is overtly upregulated in GC, both at the mRNA and protein levels.

**Fig. 6:** YAP1 mRNA expression and patient prognosis in GC, based on Oncomine and KMPLOT database analysis. DErrico Gastric Statistics in the Oncomine database revealed that YAP1 was highly expressed in GC tissues (**a**). YAP1 mRNA expression was elevated in gastric intestinal adenocarcinoma (**b**), diffuse gastric adenocarcinoma (**c**) and gastric mixed adenocarcinoma (**d**) compared with the gastric normal mucosa. KMPLOT database analysis demonstrated that patients with high YAP1 expression had poor prognosis, with shorter overall survival (**e**) and reduced first progression time (**f**) compared with the low YAP1 expression cohort

## Discussion

Although the incidence of gastric cancer has been slowly declining over the past years, it remains the second leading cause of cancer death around the world. Because of its inevitable invasiveness and metastatic potential, most GC cases are diagnosed at an advanced stage. Therefore, chemotherapy and target therapy remain the main treatment options for GC [28]. It is urgent to identify useful biomarkers and new targets for GC diagnosis and therapy.

Recent studies have demonstrated that lncRNAs might play vital roles in tumor physiological and pathological processes. LncRNAs significantly influence multiple life processes in tumor cells, by regulating cell proliferation, apoptosis, invasion and metastasis [29–31]. In the present study, we found that the novel lncRNA LATS2-AS1-001 and its neighboring gene LATS2 were downregulated in GC compared with matched normal mucosa specimens, and decreased LATS2-AS1-001 and LATS2 expression levels were related to TNM stage. In addition, there was a strong correlation between LATS2-AS1-001 and LATS, both of which could be used as diagnostic indexes in GC. Additionally, we explored the function and mechanism of LATS2-AS1-001 in GC. In vitro assays showed that LATS2-AS1-001 overexpression resulted in reduced GC cell viability and colony formation ability, and enhanced GC cell G0/G1 phase arrest. Furthermore, ectopic expression of LATS2-AS1-001 inhibited GC cell invasion and metastasis both in scratch and Transwell assays. These results suggested that LATS2-AS1-001 might act as a tumor suppressor in GC. Mechanistically, we performed qRT-PCR and Western blot to detect LATS2 and YAP1 amounts after LATS2-AS1-001 overexpression. The results showed that ectopic expression of LATS2-AS1-001 in GC cells dramatically upregulated LATS2 and induced YAP1 phosphorylation via binding to EHZ2. These results suggested that LATS2-AS1-001 could exert its tumor suppressor role by regulating LATS2 and YAP1 via binding to EZH2.

Antisense lncRNAs are identified as transcription products from the opposite strand of the protein-coding or sense strand, which contribute to corresponding gene regulation by gene silencing or via degradation of sense transcripts [31, 32]. Previous studies have shown that the tumor-related genes ADAMTS9 (ADAM metallopeptidase with thrombospondin type 1 motif 9) and MAPT are regulated by their corresponding antisense long non-coding RNAs, respectively, in glioma and ER-negative breast cancer [33, 34]. Korneev et al. [35] have shown that NATS, a long non-coding natural antisense transcript, is complementary to RNA transcripts that encode NOS1 (nitric oxide synthase 1). NATS negatively regulates NOS1 expression. Sun et al. [36] revealed that FGFR3-AS1 (FGFR3 antisense transcript 1) functions as an oncogene to promote osteosarcoma progression by upregulating FGFR3. All the aforementioned data demonstrate that natural antisense transcripts play vital roles in tumor formation and progression by regulating their corresponding sense genes [37]. The above findings suggested that antisense RNA LATS2-AS1-001 might regulate LATS2 in gastric cancer.

EZH2 functions as a regulator in human carcinomas, participating in tumor proliferation, invasion and metastasis. Recent evidence indicates that EZH2 plays a vital RNA binding role, contributing to the regulation of various lncRNAs. Xu et al. reported that lncRNA LINC-PINT inhibits melanoma cell proliferation and migration [38]. LncRNA LINC-PINT could recruit EZH2 to the promoters of its target genes (CDK1, CCNA2, AURKA and PCNA), resulting in H3K27 trimethylation and gene silencing [38]. Liu et al. found that linc01088 promotes cell proliferation via binding to EZH2 and inhibits P21 expression in non-small cell lung cancer [39]. Jin et al. demonstrated that the lncRNA MEG3 suppresses gallbladder cancer proliferation and invasion possibly via EZH2 ubiquitination. A ChIP assay revealed that lncMEG3 promotes LATS2 by directly interacting with EZH2. Indeed, EZH2 bound to the promoter of LATS2 and induced H3K27 trimethylation. Moreover, EZH2 silencing resulted in increased expression of LATS2 [40]. Other lncRNAs, such as linc00511 [41], DDX11-AS1 [42], PCAT6 [43] and AGAP2-AS1 [44], regulate LATS2 expression in multiple cancers by interacting with EZH2. Based on previous studies, we sought to confirm the interaction between EZH2 and LATS2-AS1-001 in this study. RIP confirmed that LATS2-AS1-001 bound to EZH2 in BGC823 cells. Notably, EZH2 knockdown resulted in LATS2 upregulation.

The Hippo signaling pathway is considered to be evolutionarily conserved to regulate organ size, tissue regeneration, tumorigenesis and tumor progression. It plays a vital role in tumor cell proliferation, apoptosis, invasion and metastasis. Both LATS2 and YAP1 are core components of the Hippo signaling pathway [45–47]. Once the Hippo signaling pathway is activated, MST1 and MST2 induce LATS1/2 phosphorylation; then, LATS1/2 kinases promote the binding of YAP1 to 14-3-3 proteins by phosphorylation, resulting in YAP1 inactivation and entrapment in the cytoplasm [48, 49]. Numerous studies have shown that the tumor suppressor LATS2 is downregulated in various carcinomas and that this protein impedes tumor proliferation and invasion, e.g., in GC [20], non-small cell lung cancer (NSCLC) [50, 51] and ovarian tumors [52]. Our previous studies assessed YAP1, a downstream transcriptional co-activator, which is overexpressed in gastric carcinoma and closely correlated with progression, metastasis and poor patient prognosis [25, 26]. YAP1 enhances gastric cancer proliferation, migration and invasion in vitro and in vivo. Knockdown of YAP1 significantly reduced the expression levels of LATS2-AS1-001 and LATS2 in BGC823 GC cells. Conversely, ectopic expression of YAP1 upregulates LATS2-AS1-001 and LATS2 [27]. In the present study, Oncomine and KMPLOT database analysis also demonstrated that YAP1 was highly expressed in GC tissues, and high YAP1 amounts reflected poor prognosis in GC patients. In addition, we found that LATS2-AS1-001 overexpression significantly increased LATS2 amounts and reduced YAP1 expression both at the mRNA and protein levels. These findings suggested that LATS2-AS1-001 functions as a tumor suppressor gene in GC possibly by regulating the LATS2/YAP1 signaling pathway. Therefore, we speculated that natural antisense LATS2-AS1-001 complementarily binds to LATS2 mRNA and forms a duplex RNA, subsequently modulating the frame and junction of LATS2 at the post-transcriptional level. Eventually, LATS2-AS1-001 exerts more extensive biological effects by participating in the Hippo pathway. Certainly, this hypothesis needs to be further verified in future research.

## Conclusion

In conclusion, LATS2-AS1-001 and LATS2 are lowly expressed and show a strong correlation in GC. Their expression levels are closely correlated with TNM stage, and they could be used as diagnostic indexes in GC. Moreover, LATS2-AS1-001 overexpression suppresses GC cell proliferation and progression in vitro. Mechanistically, ectopic expression of LATS2-AS1-001 increases LATS2 amounts and induces YAP1 phosphorylation via binding to EZH2. Collectively, these findings reveal that LATS2-AS1-001 may function as a tumor suppressor in GC, and may be used as a potential biomarker for GC diagnosis.
